# Needle-Free Jet Injectors' Geometry Design and Drug Diffusion Process Analysis

**DOI:** 10.1155/2021/5199278

**Published:** 2021-11-08

**Authors:** Yunfei Wang, Long Yue, Lechuan Hu, Jing Wang

**Affiliations:** ^1^School of Transportation and Vehicle Engineering, Shandong University of Technology, Zibo 255000, China; ^2^School of Energy and Power Engineering, Shandong University, Qingdao 266237, China; ^3^School of Clinical Medicine, Qilu Medical University, Zibo 255300, China

## Abstract

In order to study the injection and diffusion process of the drug in the subcutaneous tissue of a needle-free jet injectors (NFJIs) in detail and understand the influence of different nozzle geometry on the diffusion process of the drug, in this paper, numerical simulations were performed to study the diffusion process of the drug in the subcutaneous tissue of NFJIs with cylindrical nozzle. On this basis, the differences of the drug diffusion process with different nozzle geometries were analyzed. The results show that the drug diffused in the shape of ellipsoid in the subcutaneous tissue. The penetration of the drug into the subcutaneous tissue is deeper under the condition of conical nozzle and conical cylindrical nozzle at the same time. However, it takes longer to spread to the interface between skin and subcutaneous tissue in reverse.

## 1. Introduction

There are many problems with hypodermic needles injection, such as skin induration at the injection site, difficult to dispose of the waste of the injection device, and people's desire for needle-free jet injectors is increasing day by day. Needle-free jet injectors were first used for insulin injection in 1941 [1]. They use a high-velocity jet stream to puncture the skin and deposit drugs in the subcutaneous tissue. In recent years, the needle-free jet injectors have been continuously improved, and the injection effect has been greatly improved.

At present, the most representative needle-free jet injectors in the world were Intraject designed by the British Weston Medical Company and Injex of the American Equidyne company [2]. Baxter and Mitragotri [3–5] studied the relationship between penetration of the drug into the subcutaneous and jet velocity and diameter of needle-free jet injectors, and the results show that the degree of injection completeness depends on the jet diameter and the jet velocity. Zeng et al. [6] studied on the effect of different nozzle diameter on injection effect. It was found that the diffusion effect of the drug in the subcutaneous tissue was the best when the nozzle diameter was 0.3 mm. Rim et al. [7] studied the diffusion process of drug, which played a key guiding role for the design of needle-free jet injectors. Gupta et al. [8] studied the relationship between injection pressure and pain during the injection and found that higher pressure will increase the pain of the human body. The effects of different nozzle geometries on jet velocity and turbulence intensity are studied by LI et al. [9]. It was found that the length of the cylinder in the middle of the nozzle has a great influence on the average injection velocity and average turbulence intensity. Chen et al. [10] established a mathematical model for the injection process of needle-free jet injectors. The results show that with the increase of jet diameter and jet velocity, the depth of jet puncture hole will increase accordingly. Zhang et al. [11] studied the influence of the nozzle geometries of the piezoelectric needle-free syringe on the shape of the drug jet. When the nozzle geometry is cone column, a symmetrical jet with good controllability can be obtained.

The nozzle is one of the main components of the needle-free jet injectors. At present, the research on the influence of the nozzle geometries of the needle-free jet injectors on the drug diffusion process is not comprehensive. In this paper, taking the needle-free jet injectors with cylindrical nozzle as the prototype, the diffusion process of the drug into the skin was studied by numerical simulation. On this basis, nozzle geometry was modified, and the differences of drug diffusion process under different nozzle geometry conditions were compared and analyzed, so as to provide theoretical reference for the improved design of needle-free jet injectors.

## 2. Simulation Model of NFJIs

The cylindrical nozzle needle-free jet injector is selected as the prototype, because the actual injection and drug diffusion region are axisymmetric; so, the numerical simulation domain can be simplified to a two-dimensional region. The model simplification and grid diagram are shown in Figure 1 (one for every five grid points). In the figure, ABHI is the area of the nozzle, the radius of the nozzle is 0.125 mm, and the length of AB is 7 mm. The total skin thickness (CE) is 30 mm. According to the research results of a large number of literatures, a hole of equal diameter penetrating the skin will be formed in the first stage of drug injection, that is, the BJKGH region, and the total thickness is 3 mm. The BJ is the domain of epidermis and dermis, and the length of BJ is 1.67 mm. JK is located in the subcutaneous tissue with a length of 1.43 mm. DEFGKJ is the subcutaneous tissue region, and the subcutaneous tissue is the main area of drug diffusion. It is simplified to porous media in numerical simulation. The computing domain is divided into grids by ICEM, and the total number of grids is about 107000. For qualitatively analysis, in the effects of different nozzle structures on drug injection and diffusion in the subcutaneous tissue, the wall of the syringe nozzle is assumed smooth and undeformed.

At the initial time of the calculation, the medium of the nozzle, the equal diameter pore and the internal area of the skin porous media are air, and the drug solution is liquid. Considering that the liquid phase and gas phase are mixed during the injection process, the VOF model is used to calculate the two-phase flow. The porosity of the porous media area is 0.2, and the internal resistance coefficient is 200. The viscous resistance coefficients in the *x* and *y* directions are 6 × 10^11^ and 4 × 10^11^, respectively.

## 3. Analysis of Drug Diffusion Process with Cylindrical Nozzle

When the jet velocity is 160 m/s, the diffusion process of the needle-free jet injectors with cylindrical nozzle in the subcutaneous tissue is shown in Figure 2. The drug passes through a cylindrical nozzle to form a high-speed jet, which touches the surface of the skin and penetrates it. With the increase of injection volume, the drug converges at the end of the puncture hole and then spreads around with the end of the hole as the center, and the diffusion shape is approximately ellipsoidal. In addition, the diffusion center of the drug in the subcutaneous tissue gradually moved to the interface between the skin and the subcutaneous tissue over time.

The transient results of the distribution of drug were analyzed when the injection time was 4.6 × 10^−3^ s. The change of drug velocity on the center line of the nozzle is shown in Figure 3. It can be seen from the figure, before the drug touches the skin, the flow rate in the cylindrical nozzle increases gradually from 160 m/s to 205 m/s. Because of the influence of fluid viscosity, a boundary layer is formed near the wall of the nozzle, and the velocity of the drug in the boundary layer is low. As the flow rate remains constant, the velocity of the drug in the center of the nozzle increases. When the drug flows from the exit of the nozzle to the then continues to spread to the subcutaneous tissue from the end of the puncture hole. Due to the high resistance in the porous media, the flow rate decreases rapidly until it goes to zero.

In order to study the diffusion process of the drug in the subcutaneous tissue more accurately, the velocity of the drug at different skin depths at *t* = 4.6 × 10^−3^ s is shown in Figure 4. It can be seen from the figure that the maximum flow rate of the drug is located at the exit of the nozzle, and the flow rate of the drug at different injection depths decreases continuously with the *y* direction,and decreases slowly in the range of 0 ~ 0.12 mm, but decreases rapidly after *y* = 0.12 mm. According to the calculation, the Reynolds number of the liquid in the tube is 4 × 10^4^, which means that the flow state is turbulent.

## 4. Effect of Nozzle Geometry on Drug Diffusion Process

The better nozzle geometry can not only improve the effect of injection but also reduce energy dissipation and energy loss. This section will compare and analyze the diffusion process of the drug in the subcutaneous tissue under the results of conical nozzle and conical cylindrical nozzles. The geometry of the conical nozzle is relatively simple, and the key parameter is the shrinkage angle, which will increase the drug flow resistance if the shrinkage angle is too large. Due to the existence of a certain length of exit cylinder, the conical cylindrical nozzle can improve the stability of high-speed jet. The geometry diagrams of nozzles are shown in Figure 5, and the geometry parameters of each type of nozzle are given in Table 1.

The inlet velocity of all examples is 160 m/s. When the injection time *t* = 4.6 × 10^−3^ s, the variation of drug volume fraction with injection depth is shown in Figure 6. When the nozzle geometry is cylindrical, the diffusion depth of the drug in the subcutaneous tissue is about 7.2 mm, while for the conical nozzle and conical cylindrical nozzle, the diffusion depth is about 7.8 mm, which is larger than that of the cylindrical nozzle.

The reason for this phenomenon is conical nozzle and conical cylindrical nozzles have smaller outlet diameters. The speed of the drug in the middle of the outlet is greater; so, the penetration depth is greater at the same time. The diffusion of the drug in the subcutaneous tissue with different nozzle geometries is shown in Figure 7. Compared with Figure 2, when the drug just flow out of the puncture hole, there is a large difference in the diffusion morphology of the drug in the subcutaneous tissue. With the passage of time, the diffusion form of the drug is roughly the same, and it spreads around in the form of ellipsoid. At the time of *t* = 1.2 × 10^−3^ s, the drug of the cylindrical nozzle has reached the interface between the skin and subcutaneous tissue and diffused in all directions on the interface (as shown in Figure 2(e)). For the conical and the conical cylindrical nozzle, the drug has not fully reached the interface between the skin and subcutaneous tissue, which is due to the higher speed of the drug entering the subcutaneous tissue, the deeper depth of the skin at the same time. So, it takes longer to spread to the interface between skin and subcutaneous tissue in reverse. In addition, according to Figures 7(c) and 7(f), it can be judged that the drug diffuses outward as an ellipsoid in the subcutaneous tissue, and the closer it is to the interface between the skin and subcutaneous tissue, the smaller the volume fraction of the drug.

The diffusion distances of the drug at different depths in the subcutaneous tissue along the *y*-axis positive direction at the time of *t* = 4.6 × 10^−3^ s are shown in Figure 8. As can be seen from the figure that the diffusion distance of cylindrical nozzle in *y*-axis positive direction is larger at an injection depth of less than 4 mm, the diffusion distance of conical and the conical cylindrical nozzle along *y*-axis positive direction is similar. The diffusion depth along the *y*-axis positive direction increases with the increase of the depth in the *x* direction, but it is all smaller than that of the cylindrical nozzle. When the injection depth is greater than 4 mm, the diffusion distance of drug of the conical nozzle and conical cylindrical nozzle along the *y*-axis positive direction is higher than that of cylindrical nozzles. Then, the diffusion distance decreases with the increase of depth from skin until it decreases to zero.

## 5. Conclusions

In this paper, numerical simulations were performed to study the diffusion process of the drug in the subcutaneous tissue of NFJIs with cylindrical nozzle, and the differences of the drug diffusion process with different nozzle geometries were analyzed. The following conclusions were obtained.

1. The diffusion rate of the drug decreases rapidly in the process of diffusion in the subcutaneous tissue, and the shape of diffusion is similar to ellipsoid
2. Due to the obvious increase of the velocity of drug at the exit of the conical nozzle and the conical cylindrical nozzle, the penetration of the drug into the subcutaneous tissue is deeper with conical nozzle and conical cylindrical nozzle at the same time. However, it takes longer to spread to the interface between skin and subcutaneous tissue in reverse
3. After the drug flows out of the cylindrical nozzle, the diffusion distance along the direction perpendicular to the axis of the nozzle decreases with the increase of depth in the subcutaneous tissue, while for conical nozzle and conical cylindrical nozzle, the diffusion distance shows a trend of increasing at first and then decreasing

## Figures and Tables

**Figure 1:** Model simplified schematic diagram.

**Figure 2:** Changes of drug volume fraction in the subcutaneous tissue. (a) Time = 4 × 10^−5^ s. (b) Time = 6 × 10^−5^ s. (c) Time = 2.1 × 10^−4^ s. (d) Time = 6 × 10^−4^ s. (e) Time = 1.2 × 10^−3^ s. (f) Time = 4.6 × 10^−3^ s.

**Figure 3:** Velocity distribution on the symmetry axis.

**Figure 4:** Comparison of velocity changes at different injection depths.

**Figure 5:** Geometry diagrams of nozzles.

**Figure 6:** Changes of drug volume fraction with depth in the subcutaneous tissue.

**Figure 7:** Comparison of drug diffusion process with different nozzle geometries. (a) *t* = 6 × 10^−5^ s, conical nozzle. (b) *t* = 2.1 × 10^−4^ s, conical nozzle. (c) *t* = 1.2 × 10^−3^ s, conical nozzle. (d) *t* = 6 × 10^−5^ s, conical cylindrical nozzle. (e) *t* = 2.1 × 10^−4^ s, conical cylindrical nozzle. (f) *t* = 1.2 × 10^−3^ s, conical cylindrical nozzle.

**Figure 8:** Change of volume fraction of drug with *y* direction.

**Table 1:** Geometry parameters of nozzles.

Geometry parameters	Symbol	Values
Inlet diameter	*d*_1_	0.25 mm
Outlet diameter	*d*_2_	0.125 mm
Contraction angle	*α*_1_	10°
Contraction angle	*α*_2_	30°
Cylinder length of exit	*L*	1 mm

## Data Availability

All data included in this study are available upon request by contact with the corresponding author (Wang Yunfei).
